The article "Preparation, optimization, and in vivo evaluation of an inhaled solution of total saponins of Panax notoginseng and its protective effect against idiopathic pulmonary fibrosis" was published in 2020. Journal: Drug Deliv.

# Preparation, optimization, and *in vivo* evaluation of an inhaled solution of total saponins of *Panax notoginseng* and its protective effect against idiopathic pulmonary fibrosis

**DOI:** 10.1080/10717544.2020.1856222

**Published:** 2020-12-13

**Authors:** Mengjiao Liu, Tianyi Zhang, Chen Zang, Xiaolan Cui, Jianliang Li, Guohua Wang

**Affiliations:** Institute of Chinese Materia Medica, China Academy of Chinese Medical Sciences, Beijing, China

**Keywords:** Total saponins of *Panax notoginseng* inhalation solution (TIS), idiopathic pulmonary fibrosis (IPF), atomization characteristics

## Abstract

Idiopathic pulmonary fibrosis (IPF) is a chronic and progressive pulmonary disease that can cause fibrotic remodeling of the surrounding lung, thus leading to respiratory failure. Although IPF is the most common form of idiopathic interstitial pneumonia, the precise mechanisms underlying this condition remain unknown. In this study, we used total saponins of *Panax notoginseng* inhalation solution (TIS) to induce idiopathic bleomycin-induced pulmonary fibrosis in rats. The uniformity of delivery dose was investigated by analyzing the aerodynamic particle size distribution and drug stability. The potential of hydrogen potential of hydrogen (pH) of the inhalation solution was 7.0 and the solvent 0.9% NaCl solution, thus meeting physiological requirements for pulmonary drug administration. The delivery rate was 1.94 ± 0.16 mg·min^−1^ and the total dose was 17.40 ± 0.04 mg. TIS was composed of five key components: notoginsenoside R_1_, ginsenosides Rg_1_, ginsenosides Re, ginsenosides Rb_1_, and ginsenosides Rd. The mass median aerodynamic diameter (MMAD) for these five components were 3.62 ± 0.05 µm, 3.62 ± 0.06 µm, 3.65 ± 0.10 µm, 3.62 ± 0.06 µm, and 3.61 ± 0.05 µm, respectively. Fine particle fraction (FPF) was 66.24 ± 0.73%, 66.20 ± 0.89%, 66.07 ± 1.42%, 66.18 ± 0.79%, and 66.29 ± 0.70%, respectively. The MMAD for inhalation solutions needs to be 1–5 µm, which indicates that the components of TIS are suitable for inhalation. It is important to control the particle size of targeted drugs to ensure that the drug is delivered to the appropriate target tissue. *In vitro* experiments indicated that TIS exhibited high rates of deposition in lung tissue, thus indicating that pulmonary delivery systems may represent a good therapeutic option for patients.

## 1. Introduction

Idiopathic pulmonary fibrosis (IPF) is a specific form of fibrosing interstitial lung disease (ILD) that is chronic and progressive. Although IPF is the most common form of idiopathic interstitial pneumonia and is associated with a poor prognosis, the precise mechanisms underlying this condition have yet to be elucidated (Hamer et al., 2020). The incidence of IPF increases annually and has been associated with living and occupational environments, the action of certain medications, inappropriate treatments, and a variety of other factors (Hutchinson et al., 2015). A number of pathological changes are known to occur in the lungs following pulmonary fibrosis: the lungs take on a bosselated and cobblestone appearance on the pleural surface, and the lung tissue becomes enlarged and fibrotic in localized areas (Wolters et al., 2014). There are significant pathological and abnormal changes when fibrotic lungs are compared with normal pulmonary fibroblasts and extracellular matrix (Richeldi et al., 2017). The diagnosis of IPF is complex but needs to consider clinical, imaging, and histological criteria (Lynch et al., 2018). Patients with IPF may have other complications and comorbidities that could affect the treatment during the clinical course of IPF. However, only a limited number of drugs are available for patients with mild to moderate forms of IPF; the final option for patients with severe IPF is pulmonary transplantation (Lin et al., 2017; Lederer & Martinez, 2018). At present, pirfenidone and nintedanib are usually administered, either orally or intravenously, for the treatment of pulmonary fibrosis (Rogliani et al., 2016; Varone et al., 2018). However, these drugs are expensive, side effects are common, are most patients report dissatisfaction with the clinical efficacy of these treatments (Mulhall et al., 2015; Lancaster et al., 2017). Consequently, there is an urgent need to develop new drugs for the treatment of IPF.

Total saponins of *Panax notoginseng* (tPNS) are extracted from the taproots or rhizomes of *Panax notoginseng (Burk) F. H.* Chen (Sanqi in Chinese). This medicine has been applied widely in traditional Chinese medicine for hundreds of years. tPNS contains five key components: ginsenosides Rg_1_, Re, Rb_1_, Rd, and notoginsenoside R_1_ (Yang et al., 2018). tPNS exerts certain therapeutic effects on diseases on the blood system, the cardiovascular system, and the nervous system, and has specific pharmacological effects, including the inhibition of thrombosis, anti-inflammatory and anti-oxidative effects, and hepatic protection (Xie et al., 2018). In previous studies, rats and rabbits were selected as research models to investigate the application of tPNS for the treatment of anti-pulmonary fibrosis. For example, tPNS was shown to inhibit epithelial–mesenchymal transition (EMT) in alveolar epithelial cells, and enhance the degradation ability of the extracellular matrix, thus demonstrating the capability of this medicine to treat pulmonary fibrosis (Ren et al., 2015). Ginsenoside Rg_1_ was also shown to produce a curative effect on bleomycin (BLM)-induced pulmonary fibrosis in rats via the caveolin-1 and TGF-β_1_ signaling pathways (Zhan et al., 2016). PNS was also shown to reduce cardiopulmonary injury and reduce the serum levels of IL-6 and IL-8 in Japanese white rabbits (Zhang et al., 2018).

In recent years, inhalation therapy has become a commonly adopted method to deliver drugs directly to the lungs and is widely accepted as the first-line therapy for the treatment of respiratory diseases, including asthma, pneumonia, chronic obstructive pulmonary disease (COPD), and many other types of lung disease (Sbirlea, 2006). A wide range of atomizers are commercially available at present. An appropriate atomizer should be selected according to indications and the specific particle size of the atomized liquid (Haidl et al., 2016). The use of an inhalation device to deliver a specific drug is particularly suitable for elderly patients. In this study, we built upon our previous findings and selected a compression atomizer and ensured that the mean particle size of the solution to be delivered was approximately 3 mm in diameter. When designing drug delivery systems for the lungs, it is important that drug particles are deposited in large quantities in the alveolar area.

tPNS is a hydrophilic medicine and is associated with obvious first-pass effects of liver and enterohepatic circulation phenomena; these factors mean that this drug has limited bioavailability if administered orally. Although injection can ensure that drugs are delivered directly into the blood to achieve good therapeutic effect, the doses used for injection are often high; this means that many patents will show poor compliance if they require frequent injections (Usach et al., 2019). Pulmonary inhalation has unique advantages for the treatment of lung disease: first, this method ensures that drugs are released directly in the lungs; second, there is a reduced risk of the drugs being metabolized by the liver or intestine. Furthermore, the doses of inhaled drugs can be much smaller than those used for injection; drugs that are delivered systemically are often administered at high doses and are often associated with side effects (Dolovich & Dhand, 2011). When drugs are delivered directly to the respiratory tract, there is a reduced risk of systemic adverse reactions, and an increased concentration of the drug in the target area. The inhalation of drugs results in a rapid clinical effect. For example, local atomization treatment can rapidly result in a curative effect in patients with bronchial inflammation and lung disease. Many types of nebulizers are available on the market; these are easy for patients to buy and use. In addition, it is not difficult to prepare drugs for inhalation; the process can be evaluated and controlled effectively. Collectively, these factors indicate that it is very important to conduct research on drugs for aerosol inhalation and to evaluate the clinical application of such drugs (Newman, 2017; Fuglø-Mortensen et al., 2019).

In this study, we prepared inhalation solutions containing total saponins of *Panax notoginseng* inhalation solution (TIS) for pulmonary delivery in a rat model of BLM-induced pulmonary fibrosis and evaluated the effect of this treatment using a next generation impactor (NGI), a breath simulator (BRS), and a Malvern laser granulometer. We also determined a range of *in vitro* physicochemical characteristics for the TIS, including aerosol form, pH, osmotic pressure, fine particle fraction (FPF), mass median aerodynamic diameter (MMAD), and geometric standard deviation (GSD).

## 2. Materials and methods

### 2.1. Chemicals

Total saponins of *Panax notoginseng* was acquired from the National Institutes for Food and Drug Control (purity: ≥98%, batch number: 110870-201904) and the tPNS used to prepare TIS was prepared by our laboratory. Acetonitrile was purchased from Thermo Fisher Scientific (Waltham, MA). Distilled water (Watsons Co., Ltd., Guangzhou, PR China) was HPLC grade; all other chemical reagents used during this study were of analytical grade.

### 2.2. Animals

Male Sprague-Dawley rats (weighing 180–200 g) were purchased from Vital River Laboratories Company (Beijing, China). The rats were fed ad libitum with food and water in a standard laboratory and the indoor temperature was maintained at 22–25 °C. Humidity was kept constant at 60% and the photoperiod was set to 12-h light/12-h dark. All animal experiments used in the study were approved by the Academy of Chinese Medical Science’s Administrative Panel on Laboratory Animal Care and were performed in accordance with institutional guidelines and ethics as part of the China Academy of Chinese Medical Sciences (February 1 2016).

### 2.3. HPLC analysis

The components of tPNS (ginsenosides Rg_1_, Re, Rb_1_, Rd, and notoginsenoside R_1_; Figure 1) were quantitated by reverse phase HPLC (LC-20A High Performance Liquid Chromatography System (SPD-20A detector; Shimadzu Company, Kyoto, Japan)) according to the national drug standards for tPNS (CFDA, 2020b). Chromatographic separation was performed on a Diamonsil C18 column (250 mm × 4.6 mm, 5 mm) at 25 °C. The linear gradient system consisted of A (acetonitrile) and B (water). The gradient elution profile was as follows: 0–20 min, 20% A; 20–45 min, 20–46% A; 45–55 min, 46–55% A; 55–60 min, 55% A. For all five components, the signal was monitored at 203 nm. The flow rate was maintained at 1 mL/min. Re-equilibration duration was 20 min between individual runs. All collected samples were filtered through a 0.45 mm Millipore membrane filter, and the injection volume for samples was 10 μL in each experiment.

**Figure 1.** The five components of total saponins of *Panax notoginseng* inhalation solution (TIS). (A) Notoginsenoside R_1_; (B) ginsenosides Rg_1_; (C) ginsenosides Re; (D) ginsenosides Rb_1_; (E) ginsenosides Rd.

### 2.4. The feasibility of preparing TIS

#### 2.4.1. The effect of pH on the stability of TIS

First, we prepared a range of phosphate buffers (PBS) at different pH values (2.0, 5.0, 6.8, 7.0, and 8.0). Next, we placed 500 μL of 25 mg/mL tPNS aqueous solution into a 10 mL flask, added a fixed volume of PBS at different pH values, and then sealed the solution in ampoules. The ampoules were placed at 40 °C for a total period of 10 days. The composition of the tPNS was analyzed at 0, 1, 2, 5, and 10 d. The values presented represent the means of at least six determinations.

#### 2.4.2. The effect of osmotic pressure on the stability of TIS

According to a previous study, when used without an adjustment of osmotic pressure, distilled water can be strong irritant when inhaled and can readily induce coughing, thus inducing swelling of the epithelial cells in the airways (Mochizuki et al., 1999; Morice et al., 2019). Furthermore, hyperosmosis can improve the characteristics of sputum drainage (Jang & Choi, 2001). The inhalation of hypertonic saline is much safer than the inhalation of distilled water for the induction of sputum and is therefore more appropriate (Matsuura et al., 1993). However, many studies have also shown that hypotonic and isotonic fluids have little influence on sputum drainage, while hypertonic fluids induce a significant increase in airway secretion (Makris et al., 2006; Lúcia Vaz Masson & Maria de Araújo, 2018; Roodsari & Zehtabchi, 2018). The osmotic pressure of the atomized inhalation solution should have an iso-osmotic effect. Consequently, the prescription of TIS used in this study involved 0.9% sodium chloride. Hence, we used Malvern Instruments (Malvern Instruments Ltd., Worcestershire, UK) to determine whether there were any significant differences between the use of distilled water and 0.9% sodium chloride.

### 2.5. Evaluation of TIS

#### 2.5.1. Real-time particle size

Malvern Spraytec was used to monitor the particle size diameter (PSD) of aerosols. The nebulizer was filled with 2 mL of TIS and the total collection time was 5 min; this timescale was chosen as our previous studies have shown that a liquid can be completely atomized on this timescale. Data were used to calculate D10, D50, D90 values relating to mean maximal PSD; these values represent 10%, 50%, and 90% of particles, respectively. Distilled water and 0.9% sodium chloride were used as solvents. The values presented represent the means of at least three determinations.

#### 2.5.2. The uniformity of the dose delivered

All parameters refer to the relevant details of the Inhalation Preparation for a Nebulizer in Part 0111 of Volume IV of the Chinese Pharmacopoeia (ChP), 2020 edition (CFDA, 2020a). The uniformity of delivered dose (UDD) involves three components and a respiratory simulator by BRS (BRS2000, Copley Scientific, Munich, Germany). First, filter membrane A collected the delivery rate (DR) for 1 min; then filter membrane B was used to collect the total delivered dose (TDD) with filter membrane A for 10 min; finally, filter membrane C collected the total exhalation dose (TED). We used a breathing simulator (BRS2000, Copley Scientific Limited, Nottingham, UK, see Figure 2) to mimic an adult breathing pattern (15 breaths per min, tidal volume of 500 mL, and an inhalation/expiration ratio of 1:1). We also used a PARI BOY SX compression atomization inhaler (with a red core atomization cup) and a BRS2000 respiratory simulator. We also investigated whether different Nebulizer angles (upper 15°, lower 15°, upper 30°, lower 30°, partial 15°, partial 30°, and vertical) had different effects on the UDD. The DR for the five components was given in ± mg/min.

**Figure 2.** The uniformity of the delivered dose of total saponins of *Panax notoginseng* inhalation solution (TIS) when delivered by a breathing simulator (BRS2000).

#### 2.5.3. Aerodynamic particle size analysis

For this part of the analysis, we used a next generation impactor (Copley Scientific, Munich, Germany) with a cooling box at 5 °C and a Pari Boy SX nebulizer (red nozzle insert, Pari Pharma GmbH, Starnberg, Germany). Flow rate was set to 15 L·min^−1^ by a high capacity vacuum pump (HCP5, Copley Scientific Limited, Nottingham, UK). A flow controller (TPK2000, Copley Scientific Limited, Nottingham, UK) was used to measure the aerosol particle size distribution (PSD). The nebulizer was connected to a NGI which was filled with 2 mL of TIS; the aerosol collection time was set to 10 min. The drug was collected in the different parts of the NGI (inhaler, throat, all stages); the drug content collected in each part of the NGI were then analyzed by HPLC. Experiments were repeated in triplicate and a range of parameters were calculated by Copley Inhaler Testing Data Analysis Software (CITDAS) (Copley Scientific Limited, Nottingham, UK), including MMAD, FPF, and GSD.

### 2.6. The effect of tPNS treatment on bleomycin-induced lung injury and pulmonary fibrosis

#### 2.6.1. Establishment of the animal model

Previous studies have shown that a single endotracheal injection of BLM (5 mg/kg) can induce pulmonary fibrosis in rats. In brief, each rat was weighed and anesthetized with an intraperitoneal injection of 1% sodium pentobarbital. A midline incision was then made in the neck and the trachea was exposed by blunt dissection. The dose group was given an injection of BLM (Haizheng Pfizer Pharmaceutical Co., Ltd., Zhenjiang, China) into the trachea at a dose of 5 mg/kg. Rats in the sham-operation group were given a single intratracheal dose of saline.

#### 2.6.2. Experimental protocol

Rats were randomly divided into five groups (20 rats per group): a model group, a sham-operation group, a low-dose group (1.04 mg/kg tPNS with nebulizer therapy for 10 min), a middle-dose group (2.09 mg/kg tPNS with nebulizer therapy for 20 min), and a high-dose group (3.13 mg/kg tPNS with nebulizer therapy for 30 min). After atomization treatment for 14 d, 10 rats from each group were anesthetized and then euthanized; the rest carried on their treatment regimens for a total of 28 d. The lung tissue was quickly excised from euthanized rats, washed, wiped, and stored for other experiments and experimental pathology.

#### 2.6.3. Lung coefficient measurement

The lung coefficient is an index for evaluating lung edema ((lung wet weight (mg)/body weight (g))×100). All lungs were cleaned several times in ice-cold normal saline. The lungs were then wiped with filter papers and the lung coefficient was calculated. The right lungs were then taken in a frozen tube and preserved at −80 °C. The left lungs were fixed with 10% formaldehyde and preserved at room temperature. Paraffin sections were then prepared for histological examination.

#### 2.6.4. Hematoxylin and eosin (HE) and Masson’s trichrome staining

The lung tissue sections were stained with HE and Masson’s trichome stain. We then used light microscopy to evaluate the occurrence of inflammation and pulmonary fibrosis. Appropriate diagnostic terms were used according to the distribution, severity, and morphological characteristics of the lesions, and the lesions were divided into four grades: slight, mild, moderate, and severe. The total degree of lesion was determined by the overall score. Sections stained with HE section were mainly used to detect inflammatory changes while those stained with Masson’s trichrome were used to determine fibrotic changes. Representative images were acquired with a light microscopy with a ×20 objective.

### 2.7. Statistical methods

Data were analyzed using SPSS version 20.0 (IBM Corp, Armonk, NY) and all figures were created by GraphPad Prism 7 (GraphPad Software Co., Ltd., San Diego, CA). Enumeration data were expressed as (*n* (%)) and compared between groups by the Chi-squared test. Measurement data were expressed as the mean ± standard deviation and compared between groups using the *t* test.

## 3. Results

### 3.1. The effect of pH on the stability of TIS

Figure 3 shows the five components of tPNS at different pH values at 0, 1, 2, 5, and 10 d. At a pH of 2, the content of the five components decreased gradually over the 10 days. Under other neutral or alkaline conditions, the content did not change significantly, and the stability was good. Therefore, a pH of 7.0 was selected as studies have shown that the mucosa of the airways can become irritated at low pH.

**Figure 3.** The content of total saponins of *Panax notoginseng* inhalation solution (TIS) at different potential of hydrogen (pH) values (A: pH = 2; B: pH = 5.8; C: pH = 6.8; D: pH = 7; E: pH = 8) was investigated at 0, 1, 2, 5, and 10 days (mean ± standard deviation; *n* = 6; 1, 2, 5, and 10 days compared with day 0, ^#^*p*< .001; NS, no significant difference).

### 3.2. Determination of the real-time particle size distribution of two solvents (distilled water and 0.9% sodium chloride)

As shown in Figure 4 and Table 1, we found that transmission levels were high for a period of time at the beginning of the atomization process, thus indicating low levels of aerosol particles in the distilled water group and the 0.9% sodium chloride group. Transmission then decreased and leveled off; this meant that the nebulizers began to produce aerosol particles continuously and in a steady manner. Toward the end of the investigation period, the transmission values increased due to an insufficiency in aerosol particles.

**Figure 4.** An analysis of two solvents by Spraytec monitors. (A) Distilled water; (B) 0.9% sodium chloride.

**Table 1.** The results of the two solvents when used with Spraytec monitors (mean ± standard deviation, *n* = 3).

	Dx (10)	Dx (50)	Dx (90)
Distilled water	1.52 ± 0.05	3.52 ± 0.09	8.14 ± 0.43
0.9% sodium chloride	1.53 ± 0.13	3.64 ± 0.09	8.38 ± 0.39

The inlet gas velocity was calibrated at 15 L·min^–1^. D10, D50, and D90 represent maximal particle size diameter that includes 10%, 50%, and 90% of particles, respectively. Values given are the mean ± SD at least three replicates.

D50 and D90 values are commonly used parameters and relate to the highest production rates of aerosol particles generated by nebulizers. These parameters can reflect the aerosol PSD. Table 1 shows that the mean values of D10 for distilled water were 1.52 mm, D50 was 3.52 mm, and D90 was 8.14 mm; the mean values of D10 for 0.9% sodium chloride were 1.53 mm, D50 was 3.64 mm, and D90 was 8.38 mm. There were no significant differences between the two solvents in terms of D50 or D90.

### 3.3. Determination of DR, TDD, and TED

Figure 5 shows a range of parameters (DR, TDD, and TED) for tPNS delivered at different angles. This may help to guide patients about the way in which they should be treated to get the best results. The DR was 1 min for the amount of the active substance collected; there was no significant difference in DR across the angles tested, except for a lower 15°. However, when atomization time remained the same, the TDD for TIS was highest when the atomizer was vertical. The DR for the vertical angle was 1.94 ± 0.16 mg·min^−1^ while the TDD for the vertical angle was 17.40 ± 0.04 mg. In general, the nebulizer was more effective at delivering drugs when used in a normal position or with an upper angle.

**Figure 5.** Delivery rate (DR), total delivered dose (TDD), and total exhalation dose (TED) of total saponins of *Panax notoginseng* inhalation solution (TIS) at different breathing angles.

### 3.4. Determination of the aerodynamic particle size distribution

MMAD and FPF, the parameters used to calculate the respirable dose, were determined from the aerodynamic PSD obtained from the NGI. As shown in Figure 6 and Table 2, the MMADs for the five components (notoginsenoside R_1_, ginsenosides Rg_1_, ginsenosides Re, ginsenosides Rb_1_, ginsenosides Rd) were 3.62 ± 0.05 µm, 3.62 ± 0.06 µm, 3.65 ± 0.10 µm, 3.62 ± 0.06 µm, and 3.61 ± 0.05 µm. The FPFs were 66.24 ± 0.73%, 66.20 ± 0.89%, 66.07 ± 1.42%, 66.18 ± 0.79%, and 66.29 ± 0.70%. When the MMAD of an inhalation solution are is within a range of 1–5 µm, then the solution can be considered as beneficial for delivery to the alveolar region. We found that the nebulizer used in this study could successfully produce droplets within this range.

**Figure 6.** Next generation impactor (NGI) results for the five components of total saponins of *Panax notoginseng* inhalation solution, as determined by high performance liquid chromatography (HPLC) (*n* = 3).

**Table 2.** Next generation impactor (NGI) results of total saponins of *Panax notoginseng* inhalation solution (TIS) when used with the Pari Boy SX nebulizer (red nozzle insert) (mean ± standard deviation, *n* = 3).

	FPF (%)	MMAD (μm)	GSD
Notoginsenoside R_1_	66.24 ± 0.73	3.62 ± 0.05	1.93 ± 0.01
Ginsenosides Rg_1_	66.20 ± 0.89	3.62 ± 0.06	1.94 ± 0.01
Ginsenosides Re	66.07 ± 1.42	3.65 ± 0.10	1.93 ± 0.01
Ginsenosides Rb_1_	66.18 ± 0.79	3.62 ± 0.06	1.95 ± 0.00
Ginsenosides Rd	66.29 ± 0.70	3.61 ± 0.05	1.94 ± 0.01

FPF: fine particle fraction; MMAD: mass median aerodynamic diameter; GSD: geometric standard deviation.

### 3.5. Morphological analysis of lung tissue

The lung surface of the sham-operation group was smooth, pink, and elastic (Figure 7(A)). Figure 7(B) shows that the lung surface of model group was uneven and dark red, the volume was reduced, the elasticity was poor, the hardness had increased, and the surface showed nodular changes. Changes of lung volume, color, and elasticity, are shown in Figure 7(C–E); these changes were mild, and the changes in lung volume, color, and elasticity, lay between the changes exhibited by the sham-operation group and the model group. Only a few lobes were dark red; these were scattered with a small amount of punctate hemorrhage and the lobes showed a slight reduction in volume (see Figure 7).

**Figure 7.** The appearance of lung tissue in the sham-operation group (A), model group (B), low-dose group (C), middle-dose group (D), and high-dose group (E) on day 28.

### 3.6. Lung coefficient

The lung coefficient can reflect the level of BLM-induced lung injury. As shown in Figure 8, BLM resulted in a notable increase in the lung coefficient compared to that in the sham-operation group at 14 and 28 days (*p*< .001 vs. sham-operation group). Nebulizer therapy at 14 days and 28 days showed that different doses of tPNS could reduce the lung coefficient. Although the low-dose group showed a reduction in lung coefficient, this was not statistically significant. Compared to the model group at 14 days and 28 days, the middle-dose group and the high-dose group showed significant reductions in lung coefficient (*p*< .01 or *p*< .05 vs. model group).

**Figure 8.** Lung coefficient data for all treatment groups (^#^*p*< .001; *p< .01; **p< .05).

### 3.7. Histological analysis of pathological changes

Figure 9 shows sections of lung tissue at 14 days stained with HE and Masson’s trichrome stain. In the sham-operation group, the alveolar structure and the bronchial epithelium were intact; there was no obvious lymphocyte or neutrophil infiltration, and there was no obvious fibrous tissue hyperplasia. In the model group, there was evidence of infiltration by a large number of lymphocytes and neutrophils, significant proliferation of alveolar fibroblasts, a thickening of the alveolar septum, and inflammatory exudation in the alveolar cavity. The degree of pathological change in each treatment group was slightly lower than that in the model group. Obvious proliferation of fibrous tissue was evident in some animals from the model group, while obvious fibrous tissue hyperplasia was evident in some groups.

**Figure 9.** Images of lung tissue on day 14 stained with hematoxylin and eosin (HE) and Masson’s trichrome (×200) in the sham-operation group (A, a), model group (B, b), low-dose group (C, c), middle-dose group (D, d), and high-dose group (E, e).

Figure 10 shows lung tissue stained in HE. There were significant differences between the model group and the sham-operation group (model group vs. sham-operation group, *p*< .001). The lung tissue in the low-dose group, middle-dose group, and the high-dose group was significantly different from that of the model group (*p*< .01). Masson’s staining showed that there was a significant difference in lung tissue when compared between the model group and the sham-operation group (model group vs. sham-operation group, *p*< .001). However, there was no significant difference between the low-dose group and the model group. There was a significant difference in lung tissue between the two high-dose groups and the model group (*p*< .01).

**Figure 10.** Day 28 hematoxylin and eosin (HE) scores (A) and Masson’s scores (B) in the sham-operation group, model group, low-dose group, middle-dose group, and high-dose group (^#^*p*< .001; *p< .01).

Figure 11 shows HE and Masson’s trichrome staining on day 28. The structure of the lung tissue in the sham-operation group remained intact and there was no obvious fibrous tissue hyperplasia. In the model group, there was evidence of infiltration by a large number of lymphocytes and neutrophils, many of the alveolar fibroblasts had proliferated, the alveolar septum had thickened, and there was inflammatory exudation in the alveolar cavity and foam cell accumulation. The whole lung showed diffusing consolidation centered on the bronchi to the surrounding lung tissue. The basic structure of the lung was completely destroyed and lung function had been lost. Compared with the sham-operation group, normal alveoli in the two high-dose groups showed mild to moderate levels of damage. There was a slight thickening of the alveolar septum and less infiltration by inflammatory cells. Obvious proliferation of fibrous tissue was evident in the model group and obvious fibrous tissue hyperplasia was seen in some of the treatment groups.

**Figure 11.** Images of lung tissue on day 28 stained with 28-d hematoxylin and eosin (HE) and Masson’s trichrome (×200) in the sham-operation group (A, a), model group (B, b), low-dose group (C, c), middle-dose group (D, d), and high-dose group (E, e).

Figure 12 shows sections of lung tissue on day 28 stained in HE. There were significant differences in the lung tissue between the model group and the sham-operation group (model group vs. sham-operation group, *p*< .001). However, there was no significant difference between the low-dose group and the model group. There were significant differences between the model group and the middle-dose group (*p*< .01). There was a significant difference in lung tissue between the high-dose group and the model group (*p*< .05). Masson’s trichrome staining showed that there was a significant difference in lung tissue between the model group and the sham-operation group (*p*< .001), but there was also no significant difference between the low-dose group and the model group. However, there was obvious difference in the lung tissue between the two high-dose groups and the model group (*p*< .05).

**Figure 12.** Day 28 hematoxylin and eosin (HE) scores (A) and Masson’s scores (B) in the sham-operation group, model group, low-dose group, middle-dose group, and high-dose group (^#^*p*< .001; *p< .01; **p< .05).

## 4. Discussion

Pulmonary drug delivery is a potential new method for delivering drugs to the lungs, especially for traditional Chinese medicine, or polypeptide protein drugs, that need to be taken rapidly and show poor bioavailability of absorption properties when taken orally for the treatment of lung diseases. In terms of providing more efficient delivery, a breath-enhanced nebulizer (such as the Pari Boy SX, which is attached to a compressor to produce compressed gas) can deliver a more stable and consistent aerosol to the lungs when directed to the medication-holding chamber through a narrow hole, thus reducing the risk of drug waste.

United States Pharmacopoeia (USP) and ChP can contain a range of aerosol inhalation solutions; usually, the volume of these solutions is 2–3 mL and the atomization time is 10–15 min. In the present study, we considered atomization time and residual volume and determined that the volume of the atomization inhalation solution was 2 mL and that the atomization time was approximately 10 min. The pH of the atomized solution was controlled at pH 7.0 (neutral) and 0.9% NaCl solution was used to reduce stimulation. Our experiments showed that when the atomizer was used at different angles, there was a clear effect on the atomization characteristics of the inhaled solution; this may lead directly to differences in therapeutic efficacy. Therefore, our data suggest that patients should adjust the angle of their nebulizer vertically or upwards during the atomization process; this practice will facilitate drug delivery. Next, we used NGI and Spraytec to test the PSD of aerosols from nebulizers. These techniques directly determine the weights and aerodynamic particle sizes of therapeutically active pharmaceutical ingredients (APIs) and indicate the possible location of deposition within the respiratory tract. We found that the MMADs of the five components were 3.62 ± 0.05 µm, 3.62 ± 0.06 µm, 3.65 ± 0.10 µm, 3.62 ± 0.06 µm, and 3.61 ± 0.05 µm, respectively. The FPFs were 66.24 ± 0.73%, 66.20 ± 0.89%, 66.07 ± 1.42%, 66.18 ± 0.79%, and 66.29 ± 0.70%, respectively.

*In vitro* quality control is the best guarantee for aerosol inhalation preparations with regards to a good *in vivo* effect; particle size analysis is the most important quality control index (Sbirlea, 2006; Sheth et al., 2013). Controlling the particle size is highly beneficial with regards to the efficient deposition of particles in the lungs.

The effect of sodium chloride on atomization can improve aerosol formation and also the rate of atomization. When sodium chloride is not present, the air mist undergoes diffusion around the fog inlet; this is not appropriate for inhalation. Following the addition of sodium chloride, the air mist becomes columnar and the rate of atomization increased. These observations may be explained by the fact that sodium chloride could have changed the surface tension of the solution. As the concentration of sodium chloride increases, the surface tension of the solution decreases, thus making it easier to atomize and less likely to condense at the fog outlet of the atomizer (Ghazanfari et al., 2007; Qian et al., 2019).

Over recent years, the BLM-induced animal model has become the best experimental tool for studying IPF (Clark et al., 1983). In our rat models, we observed two processes to study the effect of a specific drug on the progression of pulmonary fibrosis at different time points. Various doses of tPNS were given at different atomization suction times; this allowed us to study its protective effect against IPF. After 14 days of tPNS treatment, there was a significant reduction in the lung coefficients and alveolitis scores. Alveolus inflammation was prominent on day 14 following the administration of BLM. On day 28, we observed significant fibrosis. The features of IPF induced in our animal models were consistent with those described in previous studies (Sabry et al., 2014). It was evident that aerosol inhalation could delay the development of pulmonary fibrosis, at least to a certain extent, and that the actual dose is lower than the dose applied clinically. We also found that the degree of pathological change in the lung tissue was mild, and there were no obvious adverse reactions. Consequently, this system is a safe and effective method for administering drugs.

By the end of July 2020, over 4 million people had been confirmed to be infected COVID-19 and over 200 people had died. Emerging data from the COVID-19 pandemic suggest that there could be substantial fibrotic consequences following SARS-CoV-2 infection (George et al., 2020). The development of anti-fibrosis drugs is there critically important in the prevention of fibrosis. Future studies should investigate the specific respiratory characteristics of patients with pulmonary fibrosis.

## 5. Conclusions

We investigated the effect of pH, osmotic pressure, the five components of TIS, and a range of key parameters (DR, TDD, TED, MMAD, and D50) by applying the BRS 2000 breath simulator, Spraytec, and NGI *in vitro*. Our results demonstrated that the Pari Boy SX with a red nozzle insert produced the smallest aerodynamic particle size for TIS and that this could be used to inhibit the development of IPF.
